# EEG-Based Epilepsy Recognition via Multiple Kernel Learning

**DOI:** 10.1155/2020/7980249

**Published:** 2020-09-29

**Authors:** Yufeng Yao, Yan Ding, Shan Zhong, Zhiming Cui

**Affiliations:** ^1^The Institute of Intelligent Information Processing and Application, Soochow University, Suzhou 215006, China; ^2^Department of Computer Science and Engineering, Changshu Institute of Technology, Changshu 215500, China; ^3^Suzhou University of Science and Technology, Suzhou 215009, China

## Abstract

In the field of brain-computer interfaces, it is very common to use EEG signals for disease diagnosis. In this study, a style regularized least squares support vector machine based on multikernel learning is proposed and applied to the recognition of epilepsy abnormal signals. The algorithm uses the style conversion matrix to represent the style information contained in the sample, regularizes it in the objective function, optimizes the objective function through the commonly used alternative optimization method, and simultaneously updates the style conversion matrix and classifier during the iteration process parameter. In order to use the learned style information in the prediction process, two new rules are added to the traditional prediction method, and the style conversion matrix is used to standardize the sample style before classification.

## 1. Introduction

Due to the proposal of support vector machine (SVM) [1] and the development of related theories, the kernel method has become an effective method to deal with nonlinear fractional data. Since the performance of the classification algorithm depends largely on the representation of data, the kernel method uses relatively simple functional operations to map samples to higher dimensions, avoiding the design of feature space and complex inner product calculation in feature space. For example, in [2], a fast kernel ridge regression was proposed by using the kernel method. In the last decades, the kernel method has been applied in many fields of machine learning [3–5].

However, some data sets contain samples with uneven distribution, heterogeneous features, or irregular data; the single-kernel method using only a single feature space performs poorly. And since different kernel functions have their characteristics, even in the same application, the effect of using different kernel functions may be very different, which makes the selection of kernel functions and their parameters have an important influence on the performance of the algorithm. Since one kernel function often cannot meet the requirements in some practical application scenarios, multikernel learning that combines multiple kernel functions has been attracting more attention [6].

The combination generated by multikernel learning can be the combination of the same kernel function under different parameters or the combination of many different kernel functions [7]. After years of research, compared with single kernel function, multikernel learning has stronger flexibility, higher interpretability, and better performance in data dimension reduction [8], text classification [9], domain adaptation [10], and other fields.

Although the multikernel learning algorithm fully combines the mapping ability of different kernel functions for data, essentially, it only uses the physical characteristics of samples that include similarity and distance and fails to take into account the implicit information in the stylized data set in the real situation. In practical application, in addition to the representative content information, the data set often contains a variety of style information, and samples with the same style often exist in the form of groups. For example, there are two ways of dividing the letters shown in Figure 1(a), i.e., by the content shown in Figure 1(b) and by the font shown in Figure 1(c), where each font is regarded as a style, and such data is regarded as stylized data.

To mine the style information of data, scholars have done many types of research. The second-order statistical model proposed in the literature [11] is applied to the problem of number recognition, but it only has a good effect on the data subject to the Gaussian distribution, which leads to a great limitation in the application scenario of the algorithm. The bilinear discriminant model proposed in the literature [12] has achieved good results in behavior recognition data, but the computational cost of the algorithm is relatively high. The domain Bayesian algorithm proposed in the literature [13] improves the naive Bayesian algorithm to identify the style information in the sample group, but it needs to specify a clear data distribution type for the algorithm in advance. However, the distribution of data in real situations is often complex and difficult to be determined in advance. The algorithm proposed in the literature [14, 15] uses a single mapping to mine the style information of samples and achieves excellent results in regression and classification problems, but it makes limited use of the physical characteristics of samples. The time-series style model of mining sample historical information proposed in the literature [16] and the bilayer clustering model of user's age and gender information proposed in the literature [17] effectively make use of the style information in the data in the unsupervised problem, but the algorithm is only targeted at specific fields, and the use of style information is limited.

Inspired by the above scholars, we propose style regularization least squares support vector machine based on multiple kernel learning (SR-MKL-SVM) to excavate and utilize the physical similarities between sample points and the implied style information in samples. In addition to using the physical characteristics of each basic kernel function for data mapping to express the similarity between samples, the algorithm uses the style transformation matrix to represent and mine the style information contained in the data set and takes it into the objective function. In the training process, the alternate optimization strategy is used to update the style transformation matrix in addition to the classifier parameters, and the mined style information is used to synchronously update the kernel matrix. To use the sample style information obtained by training in the process of prediction, two new prediction rules are added on top of the prediction method of traditional multikernel least squares support vector machine. Because the style information contained in the sample is used effectively in the training and prediction process, the experiments of most of the stylized data sets show that SR-MKL-SVM is relatively recent and the classical multikernel support vector machine algorithm is effective.

## 2. Related Works

### 2.1. Multikernel Learning

Let **x** and **z** be two sample vectors; *Φ* is a mapping function from the input space to the feature space. If there is a function *k*(·, ·), which can be defined as

(1) $$\begin{array}{c} k\left(x,z\right)=<\Phi \left(x\right),\Phi \left(z\right)>=\Phi^{T}\left(x\right)\Phi \left(z\right), \end{array}$$

then we call *k*(·, ·) the kernel function. Multikernel learning expects to achieve better mapping performance by combining different kernel functions. There are many ways to combine [6] kernel functions. In this study, we use the following way to find a final combined kernel function based on *M* basic kernel functions *k*_*i*_(·, ·). If we use *μ*_*i*_ to represent the kernel function coefficient, then the final combined kernel function is formulated as

(2) $$\begin{array}{c} k\left(x,z\right)=\overset{M}{\underset{i=1}{\sum }}\mu_{i}k_{i}\left(x,z\right), \end{array}$$

where

(3) $$\begin{array}{c} \overset{M}{\underset{i=1}{\sum }}\mu_{i},\;\mu_{i}>0,i=1,2,\cdots M. \end{array}$$

According to Mercer's theory, the combined kernel function generated by the above method still meets the Mercer condition.

### 2.2. Least Squares Support Vector Machine Based on Multikernel Learning

Let **D** = {(**x**_1_, *y*_1_), (**x**_2_, *y*_2_) ⋯ , (**x**_*n*_, *y*_*n*_)} be the training sample set; **x**_*j*_ ∈ **R**^*d*^ and *y*_*i*_ ∈ {+1, −1} are the label corresponding to **x**_*j*_. The objective function of the least squares support vector machine (LSSVM) proposed by Suykens [18] can be formulated as

(4) $$\begin{array}{c} \underset{w,b,\text{e}}{\min}\frac{1}{2}w^{T}w+\frac{\lambda }{2}\overset{n}{\underset{j=1}{\sum }}e_{j}^{2}\\ \text{s}.\text{t}.\;y_{j}=w^{T}\Phi \left(x_{j}\right)+b+e_{j},\;j=1,2,\cdots ,n, \end{array}$$

where **Φ**(**x**_*j*_) represents the mapped **x**_*j*_ in a high dimension, **w** and *b* are the classification hyperplane parameters, *e*_*j*_(*j* = 1, 2, ⋯*n*) is the error term, and *λ* is the regularization parameter.

The Lagrange multiplier **α** is introduced into Equation (4), and its dual form can be further obtained by the Slater constraint specification:

(5) $$\begin{array}{c} \underset{a}{\max}-\frac{1}{2}\alpha^{T}K\alpha -\frac{1}{2\lambda }\alpha^{T}\alpha +\alpha^{T}Y\\ \text{s}.\text{t}.\;\alpha^{T}I_{n}=0, \end{array}$$

where **K** ∈ **R**^*n*×*n*^ is the kernel matrix. With (11), we can obtain the following two equations,

(6) $$\begin{array}{c} \alpha ={\tilde{K}}^{-1}\left(Y-bl_{n}\right),\\ b={I_{n}}^{T}{\tilde{K}}^{-1}Y{\left({I_{n}}^{T}{\tilde{K}}^{-1}I_{n}\right)}^{-1}, \end{array}$$

where $\tilde{K}=K+I/\lambda$ and **Y** = (*y*_1_, *y*_2_, ⋯,*y*_*n*_)^*T*^.

By integrating **K** into (2) and (3), we can obtain multiple kernel least squares support vector machine (MK-LSSVM) as

(7) $$\begin{array}{c} \underset{\mu }{\min}\underset{\alpha }{\max}-\frac{1}{2}\overset{M}{\underset{i=1}{\sum }}\mu_{i}\alpha^{T}K_{i}\alpha -\frac{1}{2\lambda }\alpha^{T}\alpha +\alpha^{T}Y\\ \text{s}.\text{t}.\;\overset{M}{\underset{i=1}{\sum }}\mu_{i}=1,\;0\leq \mu_{i},\alpha^{T}l=0. \end{array}$$

Let $f\left(\mu ,\alpha \right)=\underset{\alpha }{\max}-\left(1/2\right)\sum_{i=1}^{M}\alpha^{T}K_{i}\alpha -\left(1/2\lambda \right)\alpha^{T}\alpha +\alpha^{T}Y$, and replace *f*(**μ**, **α**) with *t*; we have

(8) $$\begin{array}{c} \underset{\mu }{\min}t\\ \text{s}.\text{t}.\;f\left(\mu ,\alpha \right)\leq t,\\ {\mu l}_{n}=1,\;0\leq \mu ,\alpha^{T}l=0. \end{array}$$

It is obvious that (8) is a semi-infinite linear program (SILP) problem, which can be solved by many existing mature optimization toolkits. For an unseen sample **x**, MK-LSSVM predicts it by using the following equation:

(9) $$\begin{array}{c} y=\mathrm{sign}\left(w^{T}\Phi \left(x\right)+b\right)=\mathrm{sign}\left(\overset{n}{\underset{j=1}{\sum }}\alpha_{j}\overset{M}{\underset{i=1}{\sum }}\mu_{i}k_{i}\left(x_{j},x\right)+b\right)=\mathrm{sign}\left(\overset{M}{\underset{i=1}{\sum }}\mu_{j}\overset{n}{\underset{j=1}{\sum }}\alpha_{i}k_{i}\left(x_{j},x\right)+b\right)=\mathrm{sign}\left(\overset{M}{\underset{i=1}{\sum }}\overset{n}{\underset{j=1}{\sum }}\mu_{j}{w_{i}}^{T}\Phi_{i}\left(x\right)+b\right). \end{array}$$

### 2.3. MK-LSSVM Algorithm Process

The algorithm steps of MK-LSSVM is shown in Algorithm 1.

## 3. SR-MKL-SVM

### 3.1. Objective Function

Let **D** = {(**x**_1_^1^, *y*_1_^1^), ⋯, (**x**_1_^*t*^, *y*_1_^*t*_1_^), ⋯, (**x**_*N*_^1^, *y*_*N*_^1^), ⋯, (**x**_*N*_^*t*_*N*_^, *y*_*N*_^*t*_*N*_^)} be a training set, where the set can be divided into *N* groups according to the style. The samples in each group have the same style, and the superscript *t*_*j*_ is the number of samples in group *j*. **x**_*j*_^*k*^ ∈ **R**^*d*^(*j* = 1, 2, ⋯, *N*, *k* = 1, 2, ⋯, *t*_*j*_) is the *k*th sample in group *j*. Under the above definition, the objective function of **SR-MKL-SVM** can be formulated as

(10) $$\begin{array}{c} \underset{w_{i},b,\mu_{i},A_{j}}{\min}J_{SR-MKL-SVM}=\frac{1}{2}\overset{M}{\underset{i=1}{\sum }}\mu_{i}{w_{i}}^{T}w_{i}+\frac{\lambda }{2}\overset{N}{\underset{j=1}{\sum }}\overset{t_{j}}{\underset{k=1}{\sum }}{\left({e_{j}}^{k}\right)}^{2}+\lambda \gamma \overset{N}{\underset{j=1}{\sum }}{\left\|A_{j}^{T}-l\right\|}_{F}^{2}\\ \text{s}.\text{t}.\;y_{j}^{k}=\overset{M}{\underset{i=1}{\sum }}\mu_{i}w_{i}^{T}A_{j}^{T}\Phi_{i}\left(x_{j}^{k}\right)+b+e_{j}^{k},\\ \overset{M}{\underset{i=1}{\sum }}\mu_{i}=1,\;\mu_{i}\geq 0,i=1,2,\cdots ,M,j=1,2,\cdots ,N,k=1,2,\cdots ,t_{j}, \end{array}$$

where *μ*_*i*_(*i* = 1, 2, ⋯, *M*) is the weight coefficient of the kernel matrix, where *M* is the number of predefined kernel matrices, {**A**_*j*_ ∈ **R**^*d*×*d*^} is the style conversion matrix of the sample of style *j*, and **I** ∈ **R**^*d*×*d*^ is the identity matrix.

The first two subformulas in *J*_**SR**−**MKL**−**SVM**_ are standard MK-LSSVM expressions, and the third subformula is a penalty term using the Frobenius norm, which is used to control the degree of style conversion of the style conversion matrix to the sample, where the parameter *γ* ∈ **R**(*γ* > 0) is used. Obviously, when *γ* is larger, the deviation of the sample **A**_*j*_^*T*^*Φ*(**x**_*j*_^*k*^) is smaller after style conversion from its original style; otherwise, it is larger; especially when *γ* → +∞ is set, there is **A**_*j*_^*T*^**Φ**(**x**_*j*_^*k*^) → **Φ**(**x**_*j*_^*k*^).

### 3.2. Optimization

The goal of the algorithm is to minimize the value of *J*_**SR**−**MKL**−**SVM**_. It is very difficult to directly optimize the objective function. We can use the alternating optimization method to obtain a sufficiently available local optimal solution. When **A**_*j*_ and {**w**_*i*_, b, *μ*_*i*_} are given separately, the objective functions are optimization problems about {**w**_*i*_, b, *μ*_*i*_} and **A**_*j*_, and the above two processes are repeated until convergence or the maximum number of iterations is exceeded. To be specific,

(1) When fixing *A*_*j*_(*j* = 1, 2, ⋯, *N*), the optimization problem of formula (10) is transformed into
  (11) $$\begin{array}{c} \underset{w_{i},b,\mu_{i}}{\min}\frac{1}{2}\overset{M}{\underset{i=1}{\sum }}\mu_{i}{w_{i}}^{T}w_{i}+\frac{\lambda }{2}\overset{N}{\underset{j=1}{\sum }}\overset{t_{j}}{\underset{k=1}{\sum }}{\left(e^{k}\right)}^{2}\\ \text{s}.\text{t}.\;y_{j}^{k}=\overset{M}{\underset{i=1}{\sum }}\mu_{i}w_{i}^{T}A_{j}^{T}\Phi_{i}\left(x_{j}^{k}\right)+b+e_{j}^{k},\\ \overset{M}{\underset{i=1}{\sum }}\mu_{i}=1,\;\mu_{i}\geq 0,i=1,2,\cdots ,M,j=1,2,\cdots ,N,k=1,2,\cdots ,t_{j}. \end{array}$$
The above formula is about the standard MK-LSSVM problem of sample **A**_*j*_**Φ**_*i*_(**x**_*j*_^*k*^) after style conversion, and {*μ*_*i*_, **w**_*i*_, b} can be determined by Algorithm 1 in Section 2.2 of the article. At this time, the sample **A**_*j*_**Φ**_*i*_(**x**_*j*_^*k*^) mapped to the high dimension cannot be directly calculated, but the synthetic kernel matrix formed by the style-converted sample **A**_*j*_**Φ**_*i*_(**x**_*j*_^*k*^) can be updated by the kernel method to obtain the style-converted kernel matrix. The specific method of using the kernel method to obtain the style-converted synthetic kernel matrix will be introduced in Section 3.3 of the article
(2) When {*μ*_*i*_, **w**_*i*_, b} is fixed, then the optimization problem of Equation (10) is transformed into
  (12) $$\begin{array}{c} \underset{A_{j}\in R^{d\times d}}{\min}\frac{\lambda }{2}\overset{t_{j}}{\underset{k=1}{\sum }}{\left({e_{j}}^{k}\right)}^{2}+\lambda \gamma {\left\|A_{j}^{T}-I\right\|}_{F}^{2}\\ \text{s}.\text{t}.\;y_{j}^{k}=\overset{M}{\underset{i=1}{\sum }}\mu_{i}w_{i}^{T}A_{j}^{T}\Phi_{i}\left(x_{j}^{k}\right)+b+e_{j}^{k},\\ \overset{M}{\underset{i=1}{\sum }}\mu_{i}=1,\;\mu_{i}\geq 0,i=1,2,\cdots ,M,j=1,2,\cdots ,N,k=1,2,\cdots ,t_{j}. \end{array}$$

The above formula is a linear constrained quadratic programming problem for **A**_*j*_, which can be transformed into *N* independent problems for each **A**_*j*_ to be solved. At this time, the parameters of the synthetic kernel matrix and the classifier have been fixed, similar to the original LSSVM, and the dual form can be obtained after introducing the Lagrange multiplier to Equation (12):

(13) $$\begin{array}{c} \underset{\alpha_{j}^{k}}{\max L=}\frac{\lambda }{2}\overset{t_{j}}{\underset{k=1}{\sum }}{\left({e_{j}}^{k}\right)}^{2}+\lambda \gamma {\left\|A_{j}^{T}-I\right\|}_{F}^{2}-\overset{t_{j}}{\underset{k=1}{\sum }}\alpha_{j}^{k}\left(\overset{M}{\underset{i=1}{\sum }}\mu_{i}w_{i}^{T}A_{j}^{T}\Phi_{i}\left(x_{j}^{k}\right)+b+e_{j}^{k}-y_{j}^{k}\right)-\overset{M}{\underset{i=1}{\sum }}\left[\beta_{i}\left(1-\overset{M}{\underset{i=1}{\sum }}\mu_{i}\right)-\rho_{i}\mu_{i}\right]. \end{array}$$

Let *∂L*/*∂ ***A**_*j*_ = 0; we have

(14) $$\begin{array}{c} A_{j}^{T}=\frac{1}{2\lambda \gamma }\overset{t_{j}}{\underset{k=1}{\sum }}\overset{M}{\underset{i=1}{\sum }}\alpha_{j}^{k}\mu_{i}w_{i}\Phi_{i}^{T}\left(x_{j}^{k}\right)+I. \end{array}$$

Let *∂L*/*∂e*_*j*_^*k*^ = 0 get **α**_*j*_^*k*^ = *λe*_*j*_^*k*^. It can be seen that this formula has the same KKT [18] condition as LSSVM.

Through the process of alternating optimization, it can be known that in the process of training classifier parameters, the samples converted by the style conversion matrix are used as training data. In the first iteration, the style conversion matrix is initialized to the identity matrix. At this time, the samples after the style conversion are the same as the original samples, and no style conversion is generated. Therefore, the classifier parameters obtained by the first round of SR-MKL-SVM training are the same as the original MK-LSSVM. In the subsequent iteration process, due to the optimization of the style conversion matrix, the samples in each style group undergo the transformation of the style conversion matrix and gradually approach the standard style. The classifier parameters trained at this time fully consider the style information contained in the sample as a whole. At the same time, the process of solving the style conversion matrix from Equation (14) not only uses the physical characteristics of the samples obtained by training but also effectively uses the style information in the data. The style conversion matrix trained at this time contains each style group style information. According to the above analysis, the processes of training the classifier parameters and the style conversion matrix make full use of the style information contained in the sample, and the two processes promote each other.

### 3.3. Style Transformation

Since the dimension after the sample is mapped to the high-dimensional space may be infinite, the sample **A**_*j*_*Φ*(*x*_*j*_^*k*^) value after the style transformation cannot be obtained directly. At this point, each element in the synthetic kernel matrix can be updated with the help of the kernel method to obtain the synthetic kernel matrix after the style transformation.

Because the synthesis kernel function still has to satisfy the allowed kernel of the theorem, as *k*(**x**_*j*1_^*k*1^, **x**_*j*2_^*k*2^) = <**Φ**(**x**_*j*1_^*k*1^), **Φ**(**x**_*j*2_^*k*2^) > = ∑_*i*=1_^*M*^*μ*_*i*_*k*_*i*_(**x**_*j*1_^*k*1^, **x**_*j*2_^*k*2^), let *ϕ* be for the synthesis of the combined map of the core matrix; by formula (9), you can make the synthesis of the core matrix *k*(**x**_*j*1_^*k*1^, **x**_*j*2_^*k*2^) = <**Φ**(**x**_*j*1_^*k*1^), **Φ**(**x**_*j*2_^*k*2^) > = ∑_*i*=1_^*M*^*μ*_*i*_ < **Φ**_*i*_(**x**_*j*1_^*k*1^), **Φ**_*i*_(**x**_*j*2_^*k*2^)>; let $\hat{\Phi }\left(x_{j}^{k}\right)=A_{j}^{T}\Phi \left(x_{j}^{k}\right)$; you can get after the style conversion of the core matrix elements as

(15) $$\begin{array}{c} \hat{k}\left(x_{j1}^{k1},x_{j2}^{k2}\right)={\overset{\wedge }{\Phi }}^{T}\left(x_{j1}^{k1}\right)\hat{\Phi }\left(x_{j2}^{k2}\right)=<\hat{\Phi }\left(x_{j1}^{k1}\right),\hat{\Phi }\left(x_{j2}^{k2}\right)>=\Phi^{T}\left(x_{j1}^{k1}\right)A_{j1}A_{j2}^{T}\Phi \left(x_{j2}^{k2}\right), \end{array}$$

where $\overset{\wedge }{k}\left(x_{j1}^{k1},x_{j2}^{k2}\right)$ is the core matrix element after style transformation and **w** = ∑_*j*=1_^*N*^∑_*k*=1_^*t*_*j*_^**α**_*j*_^*k*^**Φ**(*x*_*j*_^*k*^); formula (15) can be updated to

(16) $$\begin{array}{c} \hat{k}\left(x_{j1}^{k1},x_{j2}^{k2}\right)=\Phi^{T}\left(x_{j1}^{k1}\right)A_{j1}A_{j2}^{T}\Phi \left(x_{j2}^{k2}\right)=\Phi^{T}\left(x_{j1}^{k1}\right)\cdot \left[\frac{1}{2\lambda \gamma }\overset{N}{\underset{m1=1}{\sum }}\overset{t_{m1}}{\underset{n1=1}{\sum }}\alpha_{j1}^{k1}\alpha_{m1}^{n1}\Phi \left(x_{j1}^{k1}\right)\Phi^{T}\left(x_{m1}^{n1}\right)+I\right]\cdot \left[\frac{1}{2\lambda \gamma }\overset{N}{\underset{m2=1}{\sum }}\overset{t_{m2}}{\underset{n2=1}{\sum }}\alpha_{m2}^{n2}\alpha_{j2}^{k2}\Phi \left(x_{m2}^{n2}\right)\Phi^{T}\left(x_{j2}^{k2}\right)+I\right]\cdot \Phi \left(x_{j2}^{k2}\right)=\frac{1}{4\lambda^{2}\gamma^{2}}\cdot \left[\overset{N}{\underset{m1=1}{\sum }}\overset{N}{\underset{m2=1}{\sum }}\overset{t_{m1}}{\underset{n1=1}{\sum }}\overset{t_{m2}}{\underset{n2=1}{\sum }}\alpha_{m1}^{n1}\alpha_{m2}^{n2}\alpha_{j1}^{k1}\alpha_{j2}^{k2}\cdot \langle \Phi \left(x_{j1}^{k1}\right),\left(x_{j1}^{k1}\right)\rangle \cdot \langle \Phi \left(x_{j2}^{k2}\right),\Phi \left(x_{j2}^{k2}\right)\rangle \cdot \langle \Phi \left(x_{m1}^{n1}\right),\Phi \left(x_{m2}^{n2}\right)\rangle \right]+\frac{1}{2\lambda \gamma }\overset{N}{\underset{m1=1}{\sum }}\overset{t_{m1}}{\underset{n1=1}{\sum }}\alpha_{j1}^{k1}\alpha_{m1}^{n1}\cdot \langle \Phi \left(x_{j1}^{k1}\right),\Phi \left(x_{j1}^{k1}\right)\rangle \cdot \langle \Phi \left(x_{m1}^{n1}\right),\Phi \left(x_{j2}^{k2}\right)\rangle +\frac{1}{2\lambda \gamma }\overset{N}{\underset{m2=1}{\sum }}\overset{t_{m2}}{\underset{n2=1}{\sum }}\alpha_{j2}^{k2}\alpha_{m2}^{n2}\cdot <\Phi \left(x_{j1}^{k1}\right),\Phi \left(x_{m2}^{n2}\right)>\cdot <\Phi \left(x_{j2}^{k2}\right),\Phi \left(x_{j2}^{k2}\right)>+<\Phi \left(x_{j1}^{k1}\right),\Phi \left(x_{j2}^{k2}\right)>. \end{array}$$

Because of *k*(*x*_*j*1_^*k*1^, *x*_*j*2_^*k*2^) = <*Φ*(*x*_*j*1_^*k*1^), *Φ*(*x*_*j*2_^*k*2^)> formula (16) can be updated to:

(17) $$\begin{array}{c} \hat{k}\left(x_{j1}^{k1},x_{j2}^{k2}\right)=\frac{1}{4\lambda^{2}\gamma^{2}}\cdot \left[\overset{N}{\underset{m1=1}{\sum }}\overset{N}{\underset{m2=1}{\sum }}\overset{t_{m1}}{\underset{n1=1}{\sum }}\overset{t_{m2}}{\underset{n2=1}{\sum }}\alpha_{m1}^{n1}\alpha_{m2}^{n2}\alpha_{j1}^{k1}\alpha_{j2}^{k2}\right]\cdot k\left(x_{j1}^{k1},x_{j1}^{k1}\right)\cdot k\left(x_{j2}^{k2},x_{j2}^{k2}\right)\cdot k\left(x_{m1}^{n1},x_{m2}^{n2}\right)+\frac{1}{2\lambda \gamma }\overset{N}{\underset{m1=1}{\sum }}\overset{t_{m1}}{\underset{n1=1}{\sum }}\alpha_{j1}^{k1}\alpha_{m1}^{n1}\cdot k\left(x_{j1}^{k1},x_{j1}^{k1}\right)\cdot k\left(x_{m1}^{n1},x_{j2}^{k2}\right)+\frac{1}{2\lambda \gamma }\overset{N}{\underset{m2=1}{\sum }}\overset{t_{m2}}{\underset{n2=1}{\sum }}\alpha_{j2}^{k2}\alpha_{m2}^{n2}\cdot k\left(x_{j1}^{k1},x_{m2}^{n2}\right)\cdot k\left(x_{j2}^{k2},x_{j2}^{k2}\right)+k\left(x_{j1}^{k1},x_{j2}^{k2}\right) \end{array}$$

### 3.4. Algorithm

The training algorithm of SR-MKL-SVM is listed as follows.

SR-MKL-SVM uses alternate optimization method to solve the problem, which can be divided into two steps. The first step is kernel matrix weight coefficient and classifier parameter optimized steps can be divided into two subprocesses, respectively, i.e., solving the kernel weight SILP problems and solving the linear programming problem of the classifier parameters for the synthesis of kernel matrix at the same time, the time complexity *O*(*M*^2^*n*^2^) and *O*(*n*), respectively. Due to *M* ≥ 1, the total time complexity can be treated as *O*(*M*^2^*n*^2^). The second step is to optimize the style-standardization matrix, and the time complexity of this step is *O*(*N*^2^*n*^2^). Therefore, the total time complexity of the algorithm training process is *O*(iter · (*M*^2^*n*^3^ + *N*^2^*n*^2^)), where *M* is the number of predefined basic kernel matrices, *N* is the total number of samples, *n* is the number of styles in the data set, and iter is the number of iterations of the algorithm.

Compared with typical MKL-SVM, the MK-SRLSSVM algorithm is in the process of training in style transformation matrix to the regularization processing style samples, but the multikernel support vector machine (SVM) algorithm in solving the basic kernel function in the process of the weight coefficient is applied to solve the need to invoke the original SVM algorithm in this paper; using the original LSSVM subspaces, the SVM training process is essential in solving quadratic programming problem and the nature of the training process of LSSVM for solving linear programming problems. Therefore, the computational complexity of SR-MKL-SVM in this step is far less than that of the typical MKL-SVM algorithm. The algorithm presented in this paper optimizes the weight coefficient by solving SILP problems, which is superior to the support vector machine algorithm that optimizes the weight coefficient by solving SDP problems or QCQP problems and is comparable to the multikernel support vector machine algorithm that uses SILP and other problems to solve the weight coefficient. Therefore, SR-MKL-SVM has the same complexity as typical support vector machine algorithms.

### 3.5. Prediction Rules

Two new prediction rules were defined based on MK-LSSVM in order to use the weight, classifier parameter {*μ*_*i*_, **w**, *b*} and the style transformation matrix *A*_*j*_(*j* = 1, 2, ⋯, *N*). Since the style of the sample may or may not appear in the training process in the practical application, two new prediction rules Rule 2 and Rule 3 are added into the traditional prediction method to deal with the two cases, respectively.

Let **X**_0_ = {**x**_0_^1^, **x**_0_^2^, ⋯, **x**_0_^*t*_0_^} be a subset of the entire testing data set in which each element has the same style, and **x**_0_^*t*_0_^ ∈ *R*^*d*^(*k* = 1, 2, ⋯*t*_0_) is a sample.

**Rule 1 .**

Traditional prediction method.

Traditional prediction methods only use weight *μ*_*i*_ and classifier parameters *w* and *b* to predict the sample **x**_0_^*k*^ in the testing data set and obtain the corresponding label *y*_0_^*k*^:

(18) $$\begin{array}{c} y_{0}^{k}=\mathrm{sign}\left[w^{T}\Phi \left(x_{0}^{k}\right)+b\right]=\mathrm{sign}\left[\overset{N}{\underset{j=1}{\sum }}\overset{L_{j}}{\underset{k=1}{\sum }}\alpha_{j}^{k}\overset{M}{\underset{i=1}{\sum }}\mu_{i}k_{i}\left(x_{j}^{k},x_{0}^{k}\right)+b\right]. \end{array}$$

**Rule 2 .**

Test sample style is known.

If the style of the test sample already exists in the training data set, the corresponding style transformation matrix acquired during the training process can be directly used to process the style transformation of the sample, so that the sample is close to the standard style. Then, the predicted label *y*_0_^*k*^ was obtained by using traditional prediction rules for the processed sample *A*_0_^*T*^*Φ*(*x*_0_^*k*^).

(19) $$\begin{array}{c} {y_{0}}^{k}=\mathrm{sign}\left[w^{T}{A_{0}}^{T}\Phi \left({x_{0}}^{k}\right)+b\right]=\mathrm{sign}\left[\overset{N}{\underset{j=1}{\sum }}\overset{t_{j}}{\underset{k=1}{\sum }}\alpha_{j}^{k}\overset{M}{\underset{i=1}{\sum }}\mu_{i}{\hat{k}}_{i}\left(x_{j}^{k},x_{0}^{k}\right)+b\right]. \end{array}$$

${\hat{k}}_{i}\left(x_{j}^{k},x_{0}^{k}\right)$ can be obtained from Section 3.3.

**Rule 3 .**

Test sample style is unknown.

If the sample group **X**_0_'s style does not exist in the training data set, to effectively make use of the style information obtained by training; based on the direct extrapolation idea, we consider the same style of the information contained in the sample group as a new style. The detailed steps are as follows:

**Step 1 .**

Obtain the temporary label *Y*_temp_ = {*y*_0_^1^, *y*_0_^2^, ⋯, *y*_0_^*t*_0_^} of testing data set **X**_0_ by using Rule 1.

**Step 2 .**

Train **X**_0_ and its temporary label *Y*_temp_ with the training data set to obtain the new weight ${\hat{\mu }}_{i}$, classifier parameter $\left\{\hat{w},\hat{b}\right\}$, and style transformation matrix *A*_0_^*T*^.

**Step 3 .**

Use $\left\{{\hat{\mu }}_{i},\hat{w},\hat{b},A_{0}^{T}\right\}$ to predict test set **X**_0_ and get the formal prediction label*Y*_0_ = {*y*_0_^1^, *y*_0_^2^, ⋯, *y*_0_^*t*_0_^}.

Since that most of the data in real scenes contain implicit or obvious style characteristics, the new prediction method added in SR-MKL-SVM takes into account the situation of known style and unknown style. The style information corresponding to the predicted samples is directly used to predict the samples with known styles. The direct extrapolation method is used to predict the unknown style samples, and the trained style information is used effectively, so the algorithm has good universality.

### 3.6. Analysis of SR-MKL-SVM

Different from SVM, which only searches for the optimal classification hyperplane according to the physical distribution of the original data, SR-MKL-SVM not only considers the physical characteristics contained in the data but also mines the style characteristics of the data. In this paper, the whole training samples are used to optimize the classifier parameters and the data sets with different styles are processed, respectively. With the advantage of multikernel learning for data mapping, the algorithm in this paper can represent and process the data containing more complex styles and make full use of the trained style information to conduct style regularization processing on the original samples in both training and testing methods, so that the data distribution after style transformation can be more easily divided. Compared with traditional SVM and SR-MKL-SVM, we find that SR-MKL-SVM can make full use of the information contained in the stylized data to improve the classification performance.

## 4. Experimental Results

### 4.1. Data

In this section, we introduce the EEG data provided by Bonn University to evaluate our proposed method. The EEG data set consists of 5 groups of samples from 2 groups, with detailed information as shown in Table 1, and randomly selected samples from each group as shown in Figure 2. As can be seen from Figure 2, the fluctuation of samples from different groups is very different. For example, the signal fluctuation of patients in group A and healthy people in group E is significantly different. The signal fluctuation of patients in group C and group E also differed greatly under different conditions.

Studies [19] showed that feature extraction of original EEG data in advance could effectively improve classification performance. In this paper, kernel principal component analysis (KPCA) [5, 20] was used to extract features from original data. In this section, the data after dimension reduction is used for experiments. As can be seen above, the number of samples in the data set is 500, the number of categories is 2, and the sample dimension is 70. Samples from the same group are considered to have the same style.

In order to verify the validity of this algorithm, different groups of data are selected to form two types of data sets. The first type of data is all styles contained in the test set exist in the training set at the same time. The second type of data is the test set has a style not found in the training set, and the details of the construction data set are shown in Table 2.

#### 4.1.1. Epileptic EEG Data Set

Data sets DS.1 and DS.2 are the first type of data; DS.3 and DS.4 are the second type of data. All data were random, and 10 experiments were conducted under the same set of parameters, averaging the results. Rule 2 and Rule 3 are used to predict the two types of data. The experimental results and parameters of all algorithms [21–32] are shown in Table 3.

From the experimental results in Table 3, it can be concluded that the decision tree algorithm in data set DS.1 has the best wave signal recognition effect, and the NLMKL algorithm in data set DS.2 has the best classification accuracy, leading all other algorithms including this algorithm. The results of this algorithm in the first two data sets are not as good as DT and NLMKL, but the difference is small.

From the above results, we can see the effectiveness and stability of the proposed algorithm in improving the accuracy of EEG signal recognition by mining and utilizing different fluctuation features contained in each group of samples.

## 5. Conclusion

In order to use the style information contained in the sample, this paper proposes a style regularization least squares support vector machine (SR-MKL-SVM) based on multicore learning. In addition to the advantage of multicore learning for the expression of physical similarity between samples, the algorithm also mines and uses the style information contained in the samples to improve the classification accuracy of the algorithm. SR-MKL-SVM takes the style information contained in the sample into the objective function, uses the style conversion matrix to standardize the sample, uses the regularization method to limit the degree of style conversion, and optimizes both the classifier parameters and the style standard during the training process conversion matrix. In addition to the traditional prediction methods, new prediction rules that can use the trained style information are added. Experiments in stylized data sets show the effectiveness and certain practicality of the algorithm.

## Figures and Tables

**Figure 1:** Example of stylistic data: (a) data set; (b) different contents; (c) different styles.

**Figure 2:** EEG data visualization.

**Algorithm 1:** Algorithm 1.

**Algorithm 2:** Algorithm 2.

**Table 1:** Description of epileptic EEG data set.

Group	Type
A	Healthy
B	
C	Patient
D	
E	

**Table 2:** Detail of experimental data sets.

Num	Training data	Testing data
DS.1	Each 50% z (A, B, E)	Other 50% (A, B, E)
DS.2	Each 50% (B, D, E)	Other 50% (B, D, E)
DS.3	Each 50% (A, C ,E)	Other 50% (A, C, E)
DS.4	Each 50% (A, C, E)	Other 50% (A, C, E)

**Table 3:** Experimental results of epileptic EEG.

Algorithm	Precision			
	DS.1	DS.2	DS.3	DS.4
simpleMKL	0.9273 (*C* = *e*^4^)	0.7920 (*C* = *e*^1^)	0.8133 (*C* = *e*^5^)	0.8013 (*C* = *e*^1^)
easyMKL	0.9520 (*λ*_*e*_ = 0.1)	0.8333 (*λ*_*e*_ = 0.8)	0.5333 (*λ*_*e*_ = 0.6)	0.7767 (*λ*_*e*_ = 0.3)
GMKL	0.9260 (*C* = *e*^0^)	0.7867 (*C* = *e*^5^)	0.7507 (*C* = *e*^−1^)	0.7973 (*C* = *e*^2^)
LMKL	0.9600 (*C* = *e*^0^)	0.8120 (*C* = *e*^3^)	0.8200 (*C* = *e*^3^)	0.8133 (*C* = *e*^−1^)
NLMKL	0.9507 (*C* = *e*^1^)	0.9493 (*C* = *e*^5^)	0.8293 (*C* = *e*^1^)	0.8480 (*C* = *e*^3^)
RBMKL	0.9413 (*C* = *e*^0^)	0.8440 (*C* = *e*^4^)	0.7787 (*C* = *e*^−1^)	0.8067 (*C* = *e*^−1^)
GLMKL	0.9413 (*C* = *e*^1^)	0.8333 (*C* = *e*^3^)	0.7627 (*C* = *e*^0^)	0.8227 (*C* = *e*^−1^)
CABMKL	0.9373 (*C* = *e*^2^)	0.8453 (*C* = *e*^2^)	0.7560 (*C* = *e*^0^)	0.8027 (*C* = *e*^1^)
NB	0.9520	0.8947	0.8067	0.7087
DT	0.9747	0.8467	0.7533	0.8120
SR-MKL-SVM	0.9503 (*λ* = *e*^−1^, *γ* = *e*^−3^)	0.9353 (*λ* = *e*^3^, *γ* = *e*^−5^*a*)	0.9153 (*λ* = *e*^−1^, *γ* = *e*^−2^)	0.9120 (*λ* = *e*^1^, *γ* = *e*^−1^)

## Data Availability

The original EEG data are available and can be downloaded from http://www.meb.unibonn.de/epileptologie/science/physik/eegdata.html.
